# Intelligent Recognition Algorithm-Based Color Doppler Ultrasound in the Treatment of Dangerous Placenta Previa

**DOI:** 10.1155/2021/9886521

**Published:** 2021-11-29

**Authors:** Xiaoxiao Zheng, Xiaoqiong Li, Jinxia Xu, Yunbo Wei

**Affiliations:** Department of Obstetrics, Huai'an Maternal and Child Health Hospital, No. 104 Renmin South Road, Huai'an 223001, Jiangsu, China

## Abstract

The study focused on the clinical diagnostic value of color Doppler ultrasound of dangerous placenta previa patients under the guidance of intelligent recognition algorithms. 58 patients with placenta previa and placenta accreta admitted to the hospital for treatment were selected as research subjects. The color Doppler ultrasound under the guidance of intelligent recognition algorithm was compared with the two-dimensional ultrasound for specificity, sensitivity, and accuracy. The color Doppler ultrasound results showed that, of the 58 patients, there were 32 cases of complete placenta previa and 26 cases of incomplete placenta previa, which were consistent with the surgical pathology results. It was found that patients with malignant placenta previa and placenta accreta had thickened placenta, disappeared posterior placental space, myometrium <2 mm, and increased incidence of cervical enlargement (*P* *<* 0.05). In conclusion, the recognition accuracy of color Doppler ultrasound under the guidance of the intelligent recognition algorithm is more than 90%, and it can effectively identify dangerous placenta previa, assisting doctors in diagnosis and treatment of dangerous placenta previa.

## 1. Introduction

Dangerous placenta previa may cause severe trauma, postpartum hemorrhage, blood clotting, etc., endangering the life of pregnant women [1]. Studies have shown that trophoblast cell invasion and dysplasia of uterine exfoliated tissue are serious causes of dangerous placenta. With the implementation of the second child policy, the number of patients with dangerous placenta previa has increased year by year [2, 3]. The maternal mortality rate is 7%, and the dangerous placenta previa is common in women with a cesarean section. There is likely to be placental implantation at the scar site of the last cesarean section. That is to say, placental villi have invaded part of the myometrium [4]. When women are at risk of dangerous placenta previa and placenta accreta, the placenta needs to be removed manually. It is the most serious complication of pregnancy, causing massive bleeding, uterine perforation, infection, and even death. Hence, early diagnosis and timely treatment are the key to improving the quality of delivery [5, 6].

Artificial intelligence [3] is a comprehensive discipline concerning control theory science, neuroscience, mathematics, information theory science, and game theory science. It is characterized by machines that can be as smart as human minds and can think and perceive like humans. Color Doppler ultrasound is a noninvasive diagnostic method. Under the guidance of electronic technology, it can detect the spatial information of the blood flow in the tested part in real time, and it can provide abundant blood circulation information. Therefore, it is highly valued clinically [7, 8]. Doppler color ultrasound has no radiation and minimizes the damage to pregnant women and fetuses. It is highly-safe, reliable, comfortable, and is easy to perform. The operator can see clear images and diagnose uterine differentiation, placenta, abnormalities, and the blood flow of pregnant women in time. Therefore, it is often used for early diagnosis of dangerous placenta previa. Malignant placenta can be detected by ultrasound in the middle and late stages of pregnancy, and active clinical treatment can reduce the risk of postpartum hemorrhage. Two-dimensional ultrasound can directly observe the shape and thickness of the placenta, the space behind the placenta, and the condition of the myometrium, and Doppler ultrasound can be used to detect blood flow signals. The main content of ultrasound diagnosis [9–11] includes (i) placenta previa; (ii) a lacuna is formed in the placenta; (iii) the placenta attaches to the thin muscle layer and disappears; (iv) placenta partly or completely disappears from the posterior placenta space; and (v) the interface between the front wall of the uterus and the back wall of the bladder. Doppler ultrasound image of malignant placenta shows (i) vortex of blood flow in the placental blood pool; (ii) turbulent flow in the blood pool; (iii) rich blood flow at the interface between the uterus and bladder; and (iv) increased blood vessels around the placenta. The Doppler color ultrasound can monitor blood flow and is sensitive to placental accreta. Su Jilian et al. reported that the sensitivity of Doppler color ultrasound for placenta was 98%, and the negative predictive value was 100%, meeting the best classification and exclusion criteria.

When it comes to ultrasonic images, great progress has been made from the manual identification of the indicator diagram to the use of computer identification and diagnosis. Traditional machine learning models can be divided into shallow learning and deep learning according to their structural levels. Most machine learning models are shallow learning, which are only effective for some simple or limited problems but are obviously at a disadvantage in the face of complex problems with large data scale. Deep learning network, with multiple hidden layers, can realize mapping transformation from low-dimensional space to high-dimensional space through multilayer nonlinear transformation and to distinguish and classify complex input data features in high-dimensional space. The intelligent recognition algorithm based on deep learning has a good clinical application effect for dealing with a large number of complex and numerous medical images.

In the study, 58 patients with severe placenta previa were selected as research subjects, and they all accepted the Doppler color ultrasound examination under the guidance of an intelligent recognition algorithm. Then, the diagnosis accuracy and sensitivity of the intelligent algorithm were investigated.

## 2. Materials and Methods

### 2.1. Research Subjects

In the study, 58 patients with dangerous placenta previa admitted to a tertiary hospital from March 2019 to September 2020 were selected as research subjects. They were aged between 30 and 46 years old, with an average of 38.29 ± 2.59 years old. The gestational period was between 34 and 40 weeks, with an average of 36.62 ± 3.11 weeks. The number of cesarean sections was 1–3, and the lower uterine incision was a transverse incision. The number of pregnancies was between 1 and 4. The diagnostic criteria for dangerous placenta previa were as follows: with a history of cesarean section and placenta previa was diagnosed prenatally.

Inclusion criteria: (i) diagnosed with dangerous placenta previa as per *Obstetrics and Gynecology*; (ii) all underwent surgical delivery and pathological examination, of singleton pregnancy; (iii) patients and their families were aware of and voluntarily joined this study and signed informed consent form.

Exclusion criteria: (i) not undergoing surgical pathological examination; (ii) cooperating with the doctor in the study. Additionally, patients with coagulation dysfunction and incomplete data were excluded.

### 2.2. Intelligent Recognition SVM Algorithm

SVM classification method is to maximize the classification margin by discovering the hyperplane in the space. However, practical problems are often nonlinear, and it is very difficult to find a hyperplane in the spatial dimension to separate data. SVM can construct the optimal classification structure hyperplane through the core function, so as to realize the linear global optimal solution.

In the study, the SVM classifier is used, and the icons extracted from the self-encoding decomposition group represent different classifications. For example, if there are *n* categories, *n* SVM classifiers can be built. For example, *x*_*i*_ represents the sample, *w* represents the weight matrix, *wj* represents the weight vector of the *j*th classifier, *b* represents the bias matrix, *bj* is the bias term of the *j*th classifier, *C* represents the penalty factor, *ξij* is the slack variable, *φ*(*xi*) has the nonlinear mapping function, and commonly, the kernel function *k(x)* replaces the mapping function *φ(x)* to simplify the mapping from the low-dimensional space to high-dimensional space. The ideal objective function can be expressed as follows.

(1) $$\begin{array}{c} min\frac{1}{2}{\left\|w_{j}\right\|}^{2}+C\sum_{i=1}^{l}\xi_{i}^{j},\\ s.t.\left(w_{j}\right)T\dot{\oint \left(x_{i}\right)}+b_{j}\geq 1-\xi_{i}^{j},ify_{i=}j,\\ \left(w_{j}\right)\dot{T}\oint \left(x_{i}\right)+b_{j}\leq -1+\xi_{i}^{j},ify_{i}\neq j,\;\xi_{i}^{j}\geq 0,\;i=1,2,\cdot \cdot \cdot ,l. \end{array}$$

By solving *N* optimization problems as equation (1), *N* decision functions are obtained, and *f* is the decision function as follows.

(2) $$\begin{array}{c} \left\{\begin{array}{c} f_{1}\left(x\right)=\left(w_{1}\right)\dot{T\oint^{}\left(x\right)+b_{1}}\\ \cdots \\ f_{n}\left(x\right)=\left(w_{n}\right)\dot{T}∳\left(x\right)+b_{n} \end{array}\right.. \end{array}$$

Substituting the test sample *iX* into equation (2) can obtain the sample value belonging to the decision function of each classifier. By selecting the classifier represented by the largest decision function value, the classification category of the sample can be identified calculated as follows:

(3) $$\begin{array}{c} class\left(x\right)=\left.arg\;max\left(w_{j}\right)\dot{T}k\left(x\right)+b_{j}\right). \end{array}$$

### 2.3. Intelligent Identification Process

Pattern recognition is the scientific identification to describe and classify research subjects. A pattern is to quantitatively and structurally describe an entity object, and a set of similar things is called a pattern class. Through pattern recognition, data are processed and analyzed in various ways and then described and classified. This recognition and classification technology transfers various feature description information of objects to the machine and automatically classifies various objects to their pattern classes.

Traditional pattern recognition methods include linear regression, nearest neighbor classification, and principal component analysis clustering algorithms. In recent years, with the development of machine learning technologies such as artificial neural networks (ANN), ANN-based learning technologies have become a worldwide research hotspot.  Figure 1 is the pattern recognition flow chart.

### 2.4. Ultrasound Examination

Color Doppler Ultrasound uses the top color Doppler ultrasound diagnosis system of Germany Siemens ACUSON Oxana series. Examination: the bladder of the patient should be full before the examination. The patient was in a supine position. The frequency of the probe for transabdominal examination is 2.5–5 MHz, and the frequency of the probe for transvaginal examination is 7–12 MHz. The patient was scanned for the position and thickness of the placenta, the echo of the placenta, the edges, borders, and thickness of the placenta, and the uterus. For patients whose placenta was at the bottom of the anterior wall, special attention should be paid to the continuity of the posterior wall and the correlation between the posterior bladder wall and the anterior uterine wall. The color ultrasound images of the placental substance and the posterior placenta were then analyzed.

Two-dimensional ultrasound examination: a two-dimensional ultrasound diagnosis and treatment instrument is used, and the frequency of the abdominal probe is set at 3.5 MHz. Before the examination, the patient was asked to drink water to keep the bladder full. The position of the placenta was determined by moving the probe to examine the fetus and its surrounding conditions and detect the distance between the placenta and the cervix, the uterine wall, the posterior wall of the bladder, the muscle layer, and the thickness of the placental implant.

### 2.5. Evaluation Index

The two-dimensional ultrasound and color Doppler ultrasound results were analyzed under the guidance of intelligent recognition algorithms. With the results of surgical examination as the “gold standard,” the sensitivity, accuracy, and specificity of two-dimensional ultrasound and color Doppler ultrasound were evaluated.

### 2.6. Statistical Methods

The data in this study were processed by SPSS21.0 software, and (x(−) ±*s*) and *n* (%) were used to represent measurement data (*t*-test) and count data (*χ*2), respectively. *P* *<* 0.05 indicated that the difference was statistically significant.

## 3. Results

### 3.1. Routine Placenta Data

All the cases were confirmed by surgery, including 15 cases of marginal placenta previa, 11 cases of partial placenta previa, and 32 cases of central placenta previa. The placenta was attached to the anterior wall in 20 cases, the posterior wall in 8 cases, the anterior and right wall in 2 cases, and the anterior and left wall in 1 case. Ultrasound showed 15 cases of marginal placenta previa, 12 cases of partial placenta previa, and 31 cases of central placenta previa, as shown in Figure 2.

### 3.2. Color Doppler Ultrasound in the Examination of Dangerous Placenta Previa

Of the 58 patients, 32 had complete placenta previa, 11 had partial placenta, and 15 had marginal placenta. 47 cases were detected by color Doppler ultrasound, and the correct rate was 81.03%. There were 41 cases correctly detected by both of the two-dimensional and Doppler color ultrasound and 5 cases incorrectly detected by both of the two methods, as shown in Figures 3 and 4.

### 3.3. Abnormal Results of Placental Attachment Examined by Color Doppler Ultrasound

Of the 58 patients, there were 27 cases of abnormal placental attachment, and color Doppler ultrasound detected 30 cases of abnormal placental attachment. The detection rate of various abnormal placental attachments using Doppler color ultrasound and two-dimensional ultrasound showed  ^*∗*^*P* > 0.05, and there was no statistically significant difference, as shown in Figure 5.

### 3.4. Examination Results of Dangerous Placenta Previa by Color Doppler Ultrasound under the Guidance of Intelligent Recognition Algorithm

The ultrasound examination results were compared with the surgical pathology results. The ultrasound examination results showed that, of 58 patients, there were 52 cases of complete placenta previa and 6 cases of incomplete placenta previa, which were consistent with the surgical pathological results. Ultrasound diagnosis detected 54 cases of placenta accreta and 4 cases without placental accreta. The specific results of the ultrasound examination are shown in Figure 6.

### 3.5. Comparison of Results of Placenta Previa of Surgical Pathological Examination and Ultrasound Examination under the Guidance of Intelligent Recognition Algorithms

Figure 7 shows the results detected by the intelligent recognition algorithm. It was noted that the intelligent recognition algorithm proposed in this study can locate the placenta previa position accurately, and the positioning result was basically similar to the manual positioning result of the doctor.

The white dotted line represented the manual positioning result of the doctor, and the red dotted line represented the positioning result of the intelligent recognition algorithm.

The results of the ultrasound examination were then compared with the postoperative pathological results. The ultrasound examination detected 38 cases of complete placenta previa and 10 cases of incomplete placenta previa, in line with surgical pathology. The ultrasound examination results showed that 39 cases had placenta accreta and 9 cases had no placenta accreta. Compared with surgical pathology results, 2 cases were missed and 2 cases were misdiagnosed (Figure 8).

### 3.6. Application of Color Doppler Ultrasound in the Diagnosis of Cicatricial Placenta Previa

Surgical results showed that, of 58 suspected patients, 50 cases had placenta previa and placenta accreta. The diagnostic accuracy rate of two-dimensional ultrasound for placenta previa and placenta accreta was 78.57% (43/58), which was lower than 94.29% (54/58) of color Doppler ultrasound, and the difference was statistically significant (*X*^2^ = 7.368, *P* = 0.007) (Figure 9).

### 3.7. Comparison of Conventional Two-Dimensional Ultrasound and Color Doppler Ultrasound Results

ROC curve analysis showed that the sensitivity and AUC of color Doppler ultrasound diagnosis were higher than those of conventional two-dimensional ultrasound, and the difference was statistically significant (^*θ*^*P* *<* 0.05) (Figure 10).

### 3.8. Features of Color Doppler Ultrasound with and without Placenta Implantation

Color Doppler ultrasound showed that dangerous placenta with placenta implantation has higher incidence of thickened placenta and loss of posterior placental space and significantly higher incidence of myometrium <2 mm and expanded cervical expanded than that without placenta implantation ( ^*∗*^*P* < 0.05), as shown in Figure 11.

### 3.9. Pregnancy Outcome

The amount of postpartum blood loss in pregnant women with placenta implantation was significantly higher than that in pregnant women without placenta implantation, with statistical significance ( ^*∗*^*P* < 0.05), as shown in Figure 12.

## 4. Discussion

Dangerous placenta previa refers to the presence or absence of placenta accreta on the basis of placenta previa. Placenta previa refers to the lower edge of the placenta away from the cervix, attached to the lower part of the uterus, or covering the cervix after 28 weeks of pregnancy [12]. According to the relationship between the placenta and the cervical foramen, placenta previa can be divided into 3 types: complete, partial, and marginal [13]. Studies have shown that compared with pregnant women without a history of cesarean section, the incidence of placenta previa in pregnant women with a history of cesarean section can increase by 5 times. Statistics show that the mortality rate of patients with malignant placenta previa can reach as high as 10%, seriously threatening the lives of pregnant women [14]. In order to reduce the mortality rate of pregnant women and improve their health, it is important to diagnose placenta previa and placenta accreta as soon as possible, so as to take timely measures to terminate the pregnancy.

For dangerous placenta previa, to diagnose placenta accreta or not before surgery has a great influence on the treatment effect [15]. Ultrasound is an economical and effective prenatal diagnosis method for malignant placenta previa. It can perform noninvasive multiangle examination and clearly show the relationship between placental thickness, fetal manifestations, and cervical and subuterine scars [5]. Furthermore, with the development of power Doppler and three-dimensional ultrasound technology, its sensitivity and specificity have been elevated. However, ultrasound cannot accurately assess the depth of placental accreta in patients with abnormal placental attachment.

At present, artificial intelligence algorithms have been widely used in the medical field [16]. Under the guidance of intelligent recognition algorithms, color Doppler ultrasound is used to detect malignant placenta previa. It is noninvasive, with high reproducibility and low cost [17–19]. Color Doppler ultrasound can be divided into transabdominal ultrasound and transperineal ultrasound. Transabdominal ultrasound is the simplest and a commonly used method. Color Doppler ultrasound images show that the posterior placenta space disappears, the placenta is thickened, and the myometrium at the placental attachment is significantly thinned. The images can effectively determine whether there is a placenta accreta, which facilitates the diagnosis of the doctor [20–22]. For those with a thick abdominal fat layer, the accuracy of abdominal ultrasound is reduced, consistent with results of Guo et al. [23]. At this time, the perineum multisection examination can fully make up for the missed detection of the cervix and lower uterus. Transperineal ultrasound can effectively identify the relationship between the placenta and myometrium. Most ultrasound images show swelling of the lower part of the uterus, enlarged cervix, placenta coverage, and abundant blood flow in the lower part of the uterus.

The combination of abdominal examination and perineal examination can complement each other to improve the accuracy of the detection of malignant placenta previa with placenta accreta [24, 25]. In patients with malignant placenta previa and placenta accreta, ultrasound can display obvious blood flow changes, such as abnormal blood flow in the placental cavity, abundant blood flow signals, placenta accreta, thinned echo zone between the uterus and placenta, the enlarged cervix, and the thinned myometrium. Color Doppler ultrasound can accurately identify whether it is complete placenta previa. Compared with the postoperative pathological results, there are a few missed and misdiagnosed cases of placenta accrete, consistent with results of Yuwen et al. [26]. For pregnant women with placental accreta, the hysterectomy rate and blood loss are higher, indicating a great impact of placental accreta on mothers. Timely prenatal ultrasound examination can quickly screen the lesions in the early stage, which assists doctors in judging the severity of the disease in a timely manner, and can provide an accurate basis for further treatment.

Limitations: this article does not discuss the situation of patients with malignant placenta previa combined with placenta accreta, which needs to be continuously explored in the clinic. Despite the high accuracy of color Doppler ultrasound, it cannot completely replace ultrasound due to the high cost. Hence, an appropriate examination method is required according to the patient's specific condition.

In conclusion, under the guidance of intelligent recognition algorithms, color Doppler ultrasound has high accuracy in the detection of malignant placenta previa and can correctly assess the severity of malignant placenta previa and placenta accreta. This study is of great significance for improving the quality of pregnancy and ensuring the safety of mothers and babies.

## Figures and Tables

**Figure 1:** Intelligent recognition process.

**Figure 2:** Placenta data of the subjects.

**Figure 3:** Color Doppler ultrasound in the diagnosis of malignant placenta previa.

**Figure 4:** Ultrasound image characteristics of dangerous placenta previa.

**Figure 5:** Abnormal results of placental attachment examined by color Doppler ultrasound ( ^*∗*^*P* *>* 0.05 indicated statistically significant difference between groups).

**Figure 6:** Ultrasound examination results.

**Figure 7:** Ultrasonic positioning of placenta previa based on the intelligent recognition algorithm.

**Figure 8:** Comparison of ultrasound results and surgical pathology results for placenta previa.

**Figure 9:** Application of color Doppler ultrasound in the diagnosis of placenta previa with placenta previa (^*θ*^*P* < 0.05 indicated that the difference between groups was statistically significant).

**Figure 10:** ROC curve analysis results of two-dimensional conventional ultrasound and color Doppler ultrasound (^*θ*^*P* < 0.05 indicated that the difference between groups was statistically significant).

**Figure 11:** Characteristics of color Doppler ultrasound with and without placenta implantation ( ^*∗*^*P* < 0.05).

**Figure 12:** Pregnancy outcomes ( ^*∗*^*P* < 0.05).

## Data Availability

The data used to support the findings of this study are available from the corresponding author upon request.
